RETRACTED

# Genetic Variations in Plasma Circulating DNA of HBV-Related Hepatocellular Carcinoma Patients Predict Recurrence after Liver Transplantation

**DOI:** 10.1371/journal.pone.0026003

**Published:** 2011-10-05

**Authors:** Jie Hu, Zheng Wang, Jia Fan, Zhi Dai, Yi-Feng He, Shuang-Jian Qiu, Xiao-Wu Huang, Jian Sun, Yong-Sheng Xiao, Kang Song, Ying-Hong Shi, Qi-Man Sun, Xin-Rong Yang, Guo-Ming Shi, Lei Yu, Guo-Huan Yang, Zhen-Bin Ding, Qiang Gao, Zhao-You Tang, Jian Zhou

**Affiliations:** 1 Liver Cancer Institute, Zhong Shan Hospital, Fudan University, Key Laboratory for Carcinogenesis and Cancer Invasion, the Chinese Ministry of Education, Shanghai Key Laboratory for Organ Transplantation, Shanghai, People's Republic of China; 2 Institute of Biomedical Sciences, Fudan University, Shanghai, People's Republic of China; 3 Shanghai Key Laboratory of Organ Transplantation, Zhongshan Hospital, Fudan University, Shanghi, People's Republic of China; Deutsches Krebsforschungszentrum, Germany

## Abstract

**Background:**

Recurrence prediction of hepatitis B virus (HBV)-related hepatocellular carcinoma (HCC) patients undergoing liver transplantation (LT) present a great challenge because of a lack of biomarkers. Genetic variations play an important role in tumor development and metastasis.

**Methods:**

Oligonucleotide microarrays were used to evaluate the genetic characteristics of tumor DNA in 30 HBV-related HCC patients who were underwent LT. Recurrence-related single-nucleotide polymorphism were selected, and their prognostic value was assessed and validated in two independent cohorts of HCC patients (*N* = 102 and *N* = 77), using pretransplant plasma circulating DNA. Prognostic significance was assessed by Kaplan-Meier survival estimates and log-rank tests. Multivariate analyses were performed to evaluate prognosis-related factors.

**Results:**

rs894151 and rs12438080 were significantly associated with recurrence (*P* = .003 and *P* = .004, respectively). Multivariate analyses demonstrated that the co-index of the 2 SNPs was an independent prognostic factor for recurrence (*P* = .040). Similar results were obtained in the third cohort (*N* = 77). Furthermore, for HCC patients (all the 3 cohorts) exceeding Milan criteria, the co-index was a prognostic factor for recurrence and survival (*P*<.001 and *P* = .002, respectively).

**Conclusions:**

Our study demonstrated first that genetic variations of rs894151 and rs12438080 in pretransplant plasma circulating DNA are promising prognostic markers for tumor recurrence in HCC patients undergoing LT and identify a subgroup of patients who, despite having HCC exceeding Milan criteria, have a low risk of post-transplant recurrence.

RETRACTED

## Introduction

Hepatocellular carcinoma (HCC) is a malignant tumor responsible for approximately 600,000–700,000 deaths worldwide and is becoming more prevalent not only in Southeast Asia and Africa, but also in western countries [1], [2]. Because of high infection rates with hepatitis B virus (HBV), 55% of world's HCC cases occur in China [3]. Despite improvements in surveillance and clinical treatment strategies, the prognosis of HCC remains dismal [4]. Tumor resection is the first treatment choice for early-stage HCC. However, recurrence and metastasis after curative resection remain the main factors that decrease survival [5]. Moreover, for patients with multifocal HCC or advanced cirrhosis, resection is not always feasible. Liver transplantation (LT) removes both tumors and underlying liver cirrhosis; therefore, it plays an important role in HCC management. However, the scarcity of liver donors has limited its clinical application. Thus, risk estimation of post-transplant tumor recurrence and metastasis is an essential element in selecting HCC patients for LT.

Hepatocarcinogenesis is characterized by accumulation of genetic alterations including chromosomal rearrangements, activation of oncogenes, and inactivation of tumor suppressor genes [6]. Our previous study demonstrated that genes favoring HCC metastasis progression are initiated relatively early in primary tumors [7]. Genomic information may provide better insights into HCC behavior and patient-directed therapy [8]–[11]. These findings compelled us to further investigate genetic variations associated with HCC recurrence and metastasis, which could be valuable for prediction of prognosis and selection of subsequent treatment. Single-nucleotide polymorphisms (SNPs) may represent the most common genetic variations in the human genome. As genetic markers, SNPs have several advantages over microsatellite sequence repeats, including abundance (one in every 750–1000 bp), stability, and suitability for high-throughput analysis [10], [12]. Microarray-based high-density SNP analysis makes a reproducible and rapid determination of genome-wide alterations possible. Some SNPs exhibit different allele frequencies between tumor and normal tissues [12]. Therefore, studies on SNPs genotyped from tumor DNA may help clarify the biological importance of genetic variations in the tumor genome. However, tumor tissue can only be obtained after surgery or from invasive biopsy.

Detection of biomarkers from peripheral blood obtained before surgery is more convenient and more applicable for prognosis prediction than from post-surgery tissue samples. Tumor-derived DNA has been detected in the plasma or serum of cancer patients [13]–[15]. A recently published study demonstrated that circulating DNA from tumor patients can be used to assess tumor dynamics [16], [17]. Thus, circulating DNA may be a good target to study, instead of DNA from tumor tissues, for its accessibility, simple manipulation, and available prognostic information before surgery [18]. Here, we detected genetic variations associated with prognosis in pretransplant plasma circulating DNA and evaluated the predictive value for post-transplant recurrence and metastasis in HBV-related HCC patients undergoing LT.

RETRACTED

## Materials and Methods

### Ethics statement

The study protocol was approved by The Research Ethics Committee of Zhongshan Hospital, Fudan University. Informed written consent was obtained according to the Declaration of Helsinki.

### Patients and specimens

The LT program of Zhongshan Hospital started in 2001. At the beginning, the indication of LT in our hospital was quite expanded (without macrovascular invasion, lymph node invasion and extrahepatic metastasis). Through the year 2007, we started to use Shanghai criteria for selecting HCC patients for LT (HCC patients with a solitary lesion < or  = 9 cm in diameter, no more than three lesions with the largest < or  = 5 cm, a total tumor diameter < or  = 9 cm without macrovascular invasion, lymph node invasion and extrahepatic metastasis [19]). The inclusion criteria for this study were as follows: 1) HBV background and distinctive HCC diagnosis by pathology; 2) full follow-up and clinicopathological data; and 3) well-preserved formalin-fixed, paraffin-embedded (FFPE) tissues or plasma samples extracted before LT. 4) without macrovascular invasion, lymph node invasion and extrahepatic metastasis. Our previous study and other literature reported that mTOR-based immumosuppression (Rapamycin) may improve the overall survival of HCC patients after LT [20], [21]. Thus, the present study excluded patients treated with mTOR-based immumosuppression and only included those patients using FK-506 (tacrolimus). Two hundred and nine patients were included in this study. All patients were received deceased donor liver transplantation. After LT, patients were followed with regular surveillance for recurrence or metastasis by chest radiograph, abdominal ultrasonogram, computed tomographic (CT) and AFP level measurement every 2 months in the first year, and at least every 3–4 months thereafter. A diagnosis of recurrence was based on typical imaging appearanceon and/or an elevated AFP level. Among the 209 patients included in the study, 91 developed HCC recurrence and 86 patients died (68 patients died of HCC recurrence and 18 died of transplantation-related complications). We use Lamivudine (100 mg/day) or Entecavir (0.5 mg/day) in combination with hepatitis B immunoglobulin (HBIG) to prevent HBV reactivation after LT. All patients were given 2400 IU HBIG intravenously in LT, followed by posttransplant 400 IU HBIG i.m. tid. until serum HBsAg became negative, and the titer of HBsAb is more than 150 IU/l. Thereafter, lamivudine or entecavir continued to use in the lifetime, and HBIG dosage was adjusted to keep the titer of HBsAb >150 IU/l.

RETRACTED

We designed our study referring to REMARK guidelines for reporting prognostic biomarkers in oncology [22]. The study design is shown in Figure 1. The clinicopathological characteristics of three cohorts of HCC patients are summarized in Table S1. Peripheral blood and FFPE tumor tissues were collected for DNA extraction (Supplemental Text S1).

**Figure 1:** Study design. Discovery Set consisted of 30 patients randomly selected from recurrence patients and non-recurrence patients. Training Set consisted of 102 consecutive patients from January 2004 to December 2006, while Validation Set comprised 77 consecutive patients from January 2007 to June 2008. Thirty tumor DNA samples randomly selected from the recurrence and non-recurrence groups were hybridized on SNP microarrays. Signatures associated with tumor recurrence were selected and validated in circulating DNA using two other independent patient cohorts.

### Microarray hybridization and genotyping

Tumor DNA was extracted from 30 FFPE tumor tissues (Discovery Set). Hybridization was performed on Affymetrix GeneChip Human Mapping SNP6.0 using the Human mapping SNP6.0 assay kit (Affymetrix Inc., Santa Clara, CA, USA). Plasma circulating DNA was genotyped using the MassARRAY system (Sequenom Inc., San Diego, CA, USA) and matrix-assisted laser desorption ionization-time of flight (MALDI-TOF) mass spectrometry (Supplemental Text S1).

### Statistical analysis

The Cochran-Armitage trend test was used to assess alleles associated with recurrence after LT. Unsupervised hierarchical clustering analysis was performed using Cluster software (version 3.0) and TreeView software (version 1.0.13). The Spearman rank test and Fisher's exact test were used to evaluate clinicopathological correlations. We used time to recurrence as the primary endpoint. Overall survival and tumor-related death were used as the secondary endpoint. Time to recurrence (TTR), Overall survival (OS) and tumor-related death were analyzed using the Kaplan–Meier method and the log-rank test. OS was defined as the interval between LT and death or the last observation. The data were censored at the last follow-up for living patients. TTR was measured from the date of LT until the detection of recurrent tumor or the last follow-up assessment. The data were censored for patients without tumor recurrence. Tumor-related death was defined as time from operation to HCC-related death. Patients alive at the end of follow-up were censored. Multivariate analysis using Cox proportional hazards model was used to evaluate prognosis-related factors. Data were analyzed using the statistical package SPSS 16.0 (SPSS Inc., Chicago, IL, USA). A statistical significance was set at *P*<.05. Receiver operating characteristic (ROC) curve analysis was used to determine the predictive value for tumor recurrence. All microarray data were registered into NCBI's Gene Expression Omnibus (GEO) database (http://www.ncbi.nlm.nih.gov/projects/geo/). (Accession number GSE29667).

RETRACTED

## Results

### Microarrays

Call rates <65% were often associated with highly degraded DNA from FFPE samples [23]. After strict quality control before hybridization, all 30 samples passed the call rate threshold of 65% (average, 74.4%; range, 72.1–78.1%) and were subjected to further analysis. Before analysis, we removed SNPs that had call rates <90%. After this filtration, 230,802 SNPs were included for further analysis. We used the Cochran-Armitage trend test to assess alleles associated with recurrence or metastasis after LT. We identified 1272 SNPs with *P*<.01, and among these, 30 SNPs demonstrated *P*<.001 (Figure S1C). Hierarchical clustering was performed based on the 1272 SNPs (Figure S2A) and the top 30 SNPs (Figure S2B). The top 30 SNPs, rather than the 1272 SNPs, could separate recurrence (high-risk group) from non-recurrence patients (low-risk group). The low-risk group had longer OS and TTR than the high-risk group (Figure S2C and 2D).

### Genotyping of plasma circulating DNA

To study the concordance between plasma circulating DNA and FFPE tumor DNA, we genotyped the top 30 SNPs in plasma circulating DNA from Discovery Set using the MassARRAY system. rs8059833 failed in PCR amplification and rs860056 was excluded because of low call rate (<90%) and finally we successfully genotyped 28 SNPs in plasma circulating DNA. Our results revealed that plasma circulating DNA and FFPE tumor DNA have a high concordance (98.2%). Plasma circulating DNA extracted from 102 patients in Training Set was genotyped for the 28 SNPs. As shown in Table S2, we calculated the allele frequencies between the recurrence and non-recurrence groups using Haploview software (vesion 4.1). We found that the minor alleles at *rs894151* and *rs12438080* were significantly associated with recurrence and metastasis in HCC patients after LT (*P* = .033 and *P* = .001, respectively. Table S2).

RETRACTED

### Clinicopathological characteristics and correlation with rs894151 and rs12438080

The two-year and four-year survival rates for Training Set (*N* = 102) were 58.6%, 48.5%, and the two-year and four-year recurrence rates were 36.3%, 45.1%, respectively. The genotype frequencies at *rs894151* were 67.6% (69/102) for *AA*, 29.4% (30/102) for *AG*, and 2.9% (3/102) for *GG*. The genotype frequencies at *rs12438080* were 47.1% (48/102) for *AA*, 47.1% (48/102) for *AC*, and 5.9% (6/102) for *CC*. Because of the low frequency of the minor allele homozygote at *rs894151* and *rs12438080* (3/102 and 6/102, respectively), we combined the heterozygote and minor allele homozygote patients as one group. We divided patients into two groups by *rs894151* (*AA* and *AG/GG*). Similarly, patients were divided into two groups by *rs12438080* (*AA* and *AC/CC*). We found that patients with *AG/GG* at *rs894151* have larger tumor sizes, increased tumor number and higher probability of microvessel invasion (*P* = .027, *P* = .012 and *P* = .038, respectively), while younger age and worse tumor differentiation were associated with *AC/CC* at *rs12438080* (*P* = .010 and *P* = .020, respectively; Table S3).

### Prognostic significance of rs894151 and rs12438080

Univariate analysis revealed that patients with *AG/GG* at *rs894151* or *AC/CC* at *rs12438080* were significantly associated with a decreased OS (*P* = .011and *P* = .038, respectively; Figure 2G and 2H) and TTR (*P* = .003 and *P* = .004, respectively; Figure 2D and 2E). Patients with more minor alleles showed shorter TTR and OS (Figure S3, Table S4 and S5). Other unfavorable predictors for OS were pre-LT treatment, tumor size>5 cm, multiple tumor nodes, and microvessel invasion (*P* = .050, *P*<.001, *P* = .003, and *P*<.001, respectively). Tumor size, tumor number, tumor encapsulation, and microvessel invasion also had prognostic significance for TTR (*P*<.001, *P* = .015, *P* = .011, and *P*<.001, respectively; Table 1). Multivariate analyses demonstrated that *rs12438080* was an independent prognostic factor for TTR (*P* = .042) rather than OS, while *rs894151* was not an independent prognostic factor for TTR or OS (*P* = .382 and *P* = .935, respectively; Table 1).

**Figure 2:** Prognostic significance assessed using Kaplan–Meier survival estimates and log-rank tests stratified by *rs894151* (D, G), *rs12438080* (E, H), and the co-index of the two factors (F, I). **A**, **B,** and **C** show the frequency distributions of genotypes in the non-recurrence and recurrence groups with the *p*-value calculated by chi-square test. *B represents a minor allele. Patients were divided into two groups by the co-index: patients with *AA* at both *rs894151*/*rs12438080* and patients with minor allele(s).

RETRACTED

**Table 1:** Univariate and Multivariate analyses of factors associated with survival and recurrence in Training Set.

	OS				TTR			
	Univariate		Multivariate		Univariate		Multivariate
Factors	HR (95% CI)	*P*	HR (95% CI)	*P*	HR (95% CI)	*P*	HR (95% CI)	*P*
Gender (male versus female)	0.669(0.241–1.855)	.440		NA	1.185(0.287–4.891)	.814		NA
Age (≥50 years versus <50 years)	0.870(0.507–1.491)	.612		NA	0.757(0.423–1.354)	.348		NA
Child-Pugh (B/C versus A)	1.291(0.725–2.299)	.385		NA	0.791(0.440–1.423)	.434		NA
Differentiation (III/IV versus I/II)	1.435(0.836–2.463)	.190		NA	1.571(0.879–2.808)	.127		NA
AFP (≥200 ng/ml versus <200 ng/ml)	0.914(0.529–1.578)	.746		NA	1.086 (0.608–1.941)	.780		NA
Encapsulation (none versus complete)	1.331(0.774–2.286)	.301		NA	2.183(1.199–3.976)	.011	1.527(0.827–2.819)	.176
Pre-LT treatment (yes versus no)	1.722(1.001–2.962)	.050	1.438(0.820–2.524)	.205	1.431(0.793–2.580)	.234		NA
Tumor size (>5 cm versus ≤5 cm)	3.369(1.821–6.234)	<.001	2.078(1.025–4.214)	.042	4.236(2.138–8.394)	<.001	2.998(1.334–6.733)	.008
Tumor number (multiple versus single)	2.439(1.352–4.401)	.003	1.566(0.800–3.065)	.190	2.150(1.159–3.988)	.015	1.131(0.538–2.379)	.746
Microvessel invasion (yes versus no)	3.495(1.862–6.562)	<.001	2.219(1.088–4.525)	.028	4.831(2.384–9.787)	<.001	2.843(1.341–6.027)	.006
*rs894151* (*AG*/*GG* versus *AA*)	2.062(1.182–3.596)	.011	1.026(0.549–1.920)	.935	2.483(1.374–4.486)	.003	1.333(0.700–2.538)	.382
*rs12438080* (*AC*/CC versus *AA*)	1.805(1.034–3.150)	.038	1.425(1.798–2.546)	.231	2.560(1.360–4.819)	.004	1.951(1.025–3.716)	.042
*rs894151*/*rs12438080* (*AB*/*BB* **^§^** versus *AA*)	3.357(1.577–7.146)	.002	2.032(0.878–4.704)	.098	5.137(2.022–13.050)	.001	2.791(1.048–7.436)	.040

Abbreviations: OS, overall survival; TTR, time to recurrence; HR, hazard ratio; CI, confidence interval; LT, liver transplantation; AFP, alpha-fetoprotein; NA, not adopted.

The prognostic significance was assessed using Kaplan-Meier survival estimates and log-rank tests. In multivariate analysis variables were adopted for their prognostic significance by univariate analysis with enter-stepwise selection (p<.05) and the co-index of rs894151/rs12438080 was analyzed when both SNPs were excluded. ^§^AB/BB represents patients with minor allele(s) at rs894151 and/or rs12438080. Pre-LT treatment, Tumor size, Tumor number, Microvessel invasion and *rs894151*/*rs12438080* were adopted for Cox analysis for OS. While, Encapsulation, Tumor size, Tumor number, Microvessel invasion and rs*894151*/*rs12438080* were adopted for Cox analysis for TTR.

RETRACTED

Chi-square tests revealed no correlation between *rs894151* and *rs12438080* (*P* = .469). To increase predicting power, we combined the two SNPs as a co-index. We divided patients into two groups using the combined index of *rs894151* and *rs12438080* (group I: patients with genotype *AA* at both *rs894151* and *rs12438080*; group II: patients with allele *G* at *rs894151* and/or *C* at *rs12438080*). Multivariate analyses demonstrated that the co-index (*rs894151*/*rs12438080*), tumor size, and microvessel invasion were independent prognostic factors for TTR (*P* = .040, *P = .*008, and *P* = .006, respectively), while tumor size and microvessel invasion were independent prognostic factors for OS (*P* = .042 and *P* = .028, respectively; Table 1).

### Validation

We validated the prognostic value of the co-index of *rs894151* and *rs12438080* in another independent cohort of 77 HBV-related HCC patients who undergoing LT (Validation Set) with results similar to those in Training Set. Patients with genotype *AA* at both *rs894151* and *rs12438080* had a longer TTR than patients with allele *G* at *rs894151* and/or *C* at *rs12438080*. In multivariate Cox proportional hazards analyses, the co-index was still an independent predictor of TTR (*P* = .001; Table S6).

### ROC analysis

ROC curve analysis were performed (*N* = 209) to evaluate the predictive power for recurrence. It showed that the predictive power of the co-index [area under the curve (AUC)  = 0.788] was significantly higher than that of *rs894151* (AUC = 0.683, *P* = 0.033), *rs12438080* (AUC = 0.679, *P* = 0.027), tumor number (AUC = 0.614, *P*<0.001) and encapsulation (AUC = 0.583, *P*<0.001). Tumor size (AUC = 0.699) and microvessel invasion (AUC = 0.717) also had lower AUC when compared with the co-index, but the differences were not reach statistical significance (*P* = 0.066 and *P* = 0.136 respectively, Figure 3 and Table S7).

**Figure 3:** The predictive ability of the co-index of *rs894151* and *rs12438080* compared with single markers and other clinical prognostic parameters by receiver operating characteristic (ROC) curves (A). The areas under the curve (AUCs) with 95% CI are shown in **B** (*p<.05, compared with the co-index). The details for AUC and 95% CI are also shown in Table S7.

### Milan criteria and the co-index of rs894151 and rs12438080

Among the 209 patients of the three cohorts, 94 met and 115 exceeded Milan criteria [24]. The Clinicopathological characteristics of patients exceeding Milan criteria were summarized in table S8. The three-year recurrent rates for patients within Milan criteria and exceeding Milan criteria were 12.3% and 67.3%. The survival rates were 83.8% and 40.6% respectively. We stratified the patients as within or beyond Milan criteria to evaluate the prognostic value of the co-index (*rs894151*/*rs12438080*). The log-rank test indicated that the co-index can be a novel predictor of recurrence regardless of Milan criteria (Figure 4A and 4D; Table 2). The co-index of the two SNPs (*rs894151*/*rs12438080*) in pretransplant plasma circulating DNA identified a subgroup of HCC patients with a low risk of post-transplant recurrence, despite having HCC beyond Milan criteria (Figure 4E). We also performed analysis of the co-index in patients within or exceeding UCSF criteria (Supplemental Text S1). The log-rank test indicated that, in patients exceeding UCSF criteria, the co-index of two SNPs was also associated with TTR and OS (Table S9). The results were similar to those in patients within UCSF (Table S10).

RETRACTED

**Figure 4:** The relationship of the co-index (*rs894151*/*rs12438080*) in patients within Milan criteria (upper panel) and exceeding Milan criteria (lower panel). Time to recurrence of the co-index (*rs894151*/*rs12438080*) in patients within Milan criteria (**A**) and exceeding Milan criteria (**D**). The prognostic significance was assessed using Kaplan-Meier survival estimates and log-rank tests. **B**, **E**, The recurrences in patients with *AA* at both SNPs were 0/44 (within Milan criteria) and 8/26 (exceeding Milan criteria). In patients with a minor allele, the recurrences were 16/50 (within Milan criteria) and 67/89 (exceeding Milan criteria). **C**, **F**, Frequency distributions of genotypes in non-recurrence and recurrence patients. The *p*-value was calculated by chi-square test.

**Table 2:** Kaplan-Meier survival estimates and log-rank tests of factors associated with TTR and OS in patients exceeding Milan criteria.

Factors	TTR		OS	
	HR (95% CI) *P*		HR (95% CI)	*P*
Pre-LT treatment (yes versus no)	1.016 (0.646–1.598)	.946	1.083 (0.675–1.737)	.741
Child-Pugh (B/C versus A)	1.178 (0.774–1.864)	.485	0.175(0.726–1.900)	.512
AFP (≥200 ng/ml versus <200 ng/ml)	1.134 (0.721–1.784)	.587	1.070(0.668–1.717)	.777
Differentiation (III/IV versus I/II)	1.245 (0.789–1.963)	.346	1.454(0.906–2.333)	.121
Encapsulation (none versus complete)	1.336 (0.844–2.115)	.216	0.817(0.510–1.311)	.403
Microvessel invasion (yes versus no)	2.975 (1.786–4.954)	<.001	2.916(1.679–5.064)	<.001
*rs894151*/*rs12438080* (*AB*/*BB* § versus *AA*)	4.238 (2.021–8.886)	<.001	3.244(1.546–6.805)	.002

§ AB/BB represents patients with minor allele at *rs894151* and/or *rs12438080*. Abbreviations: TTR, time to recurrence; CI, confidence interval; LT, liver transplantation; AFP, alpha-fetoprotein.

## Discussion

As a radical treatment for HCC, LT has many advantages over resection such as simultaneously curing HCC and the underlying cirrhosis in a single surgery. However, tumor recurrence and metastasis after LT remain the main obstacles for long-term survival. To achieve a low recurrence rate and reasonable distribution of limited donors, meticulous evaluation of the prognosis in recipients is crucial [25]. However, conventional prognostic factors for HCC patients are limited to clinicopathological parameters. Including Milan criteria, most LT indications for HCC patients focus on the tumor size, number of tumor nodules, and the absence of macroscopic vascular invasion or lymph nodes [24], [26], [27]. Efforts to identify more accurate prediction algorithms have revealed that tumor size and number are imperfect surrogates for predicting the metastatic potential of HCC [28]. Increasingly, more attention is being given to biological tumor markers for insights into HCC behavior. Studies on epigenetics [29]–[31], gene expression [32]–[35], and proteomics [36], [37] are beginning to yield potentially useful information. Schwartz et al [28] reported that analysis of allelic imbalance (AI) of nine microsatellites may extend Milan criteria without increasing tumor recurrence after LT. Wu et al [38] found *Histone Deacetylase 3* could serve as a biomarker for tumor recurrence following LT in HBV-Associated HCC. Our previous study demonstrated that overexpression of *Capn4* in HCC tissues was associated with tumor invasion and metastasis in HCC patients after LT [39]. In these studies, all the samples used were obtained from tumor tissues that were only available after surgery. Therefore, prognosis biomarker studies in preoperative plasma or serum are urgently needed.

RETRACTED

A small amount of circulating DNA can be detected in the plasma of healthy individuals. The levels of circulating DNA are elevated in cancer patients and are associated with poor prognosis [18], [40], [41]. Many studies suggested that the elevated circulating DNA of cancer patients was from apoptotic and necrotic tumor cells [18], [42]. Our previous study showed that circulating DNA extracted from the plasma of HCC patients displayed neoplastic characteristics [43]. Diehl et al [17] explored a new technology called BEAMing (beads, emulsion, amplification, and magnetics) to detect colorectal cancer-related genetic variations in circulating DNA and found that the genetic alterations could be used to monitor tumor dynamics in colorectal cancer patients undergoing surgery or chemotherapy. In this study, we tried to screen genetic variations in pretransplant plasma circulating DNA to identify promising biomarkers that are associated with tumor recurrence after LT. First, we used plasma circulating DNA for microarray hybridization, but the concentration and quantity did not meet the QC required for microarrays. Whole-genome amplification (WGA) offers new possibilities for genetic studies where limited DNA samples have been collected. We succeeded in harvesting sufficient DNA though WGA. However, the amplified plasma circulating DNA generated poor-quality array data, yielding a result similar to that in a previous report [44]. Therefore, we used FFPE tumor DNA for chip hybridization, then validated candidate SNPs in plasma circulating DNA using MALDI-TOF mass spectrometry. High concordance (98.2%) between FFPE tumor DNA and plasma circulating DNA was confirmed by our result.

RETRACTED

We identified two novel SNPs (rs894151 and rs12438080) located in 8q22 and 15q26 from plasma circulating DNA that were associated with HCC recurrence after LT and validated using another independent cohort of patients. The TTR was negatively associated with the number of minor alleles at rs894151 and rs12438080 (G at rs894151 and C at rs12438080). However, HCC is a polygenic, complex disease caused by the interaction of many genetic and environmental factors [45]. Variations in any one gene in the polygenic pathway may have a small effect on tumor progression. Therefore, we used the co-index—a combination of the two SNPs (rs894151 and rs12438080)—to increase the predictive power of SNPs. Multivariate analyses demonstrated that the co-index was an independent prognostic factor for recurrence. ROC analysis also showed that the predictive power of the co-index was more robust than that of any single SNP. To our knowledge, the present study is the first one to evaluate the prognostic value of genetic variations in pretransplant plasma circulating DNA in HCC patients undergoing LT.

The co-index of rs894151and rs12438080 was an independent prognostic factor for TTR (P = .040) but not for OS (P = .098), which may be attributed to the complexity of underlying factors for post-transplant survival. Besides HCC recurrence, other long-term problems such as immunosuppression-related and technique-related complications, as well as organ rejection, are also important prognostic factors which may cause mortality. In order to decrease the effect of these factors on survival, we used the endpoint of tumor-related death for further analysis. We found that the co-index of rs894151 and rs12438080 was an independent prognostic factor for tumor-related death (Table S11).

Previous studies reported several recurrence-associated factors for HCC patients. Nucleotide analogs may reduce the risk of HBV-related HCC development and prevent recurrence after resection [46], [47]. Active replication of HBV may initiate malignant transformation through a direct carcinogenic mechanism by increasing the probability of viral DNA insertion in or near proto-oncogenes, tumor-suppressor genes [48], [49]. However, new tumors developing from noncirrhosis liver graft need relatively long period. The main aim of administration of nucleoside analogues was to prevent function loss of liver graft, which was caused by HBV reactivation. Further studies that include a larger number of patients and a longer follow-up period are necessary to assess the benefits of nucleoside analogues for preventing long-term HCC recurrence after LT. Des-gamma-carboxyprothrombin (DCP), also known as the protein induced by vitamin K absence or antagonist II (PIVKA-II), is reported to be an effective tumor marker for HCC. This tumor marker is currently confirmed in Japan, Korea and Indonesia, while many studies have been performed worldwide. Fujiki et al [50] reported superiority of DCP and AFP over preoperative tumor size or number for predicting recurrence after living donor liver transplantation. Unfortunately, DCP detection is unavailable yet in our hospital. This restricted our ability to get the pre-LT DCP data of the studied patients. The prognostic value of the two SNPs in combination with DCP will be the next phase of our study.

RETRACTED

Milan criteria have been accepted worldwide and the outcomes of HCC patients within Milan criteria were similar to that of patients undergoing LT without HCC. However, the dichotomous yes/no nature of Milan criteria has been challenged for being too strict [27], [51], [52], some patients with tumors exceeding Milan criteria are also potentially curable by LT [26]–[28], [51], [52]. In the present study, for those patients exceeding Milan criteria, we found the co-index of rs894151 and rs12438080 also acted as a prognostic factor for recurrence (P<.001; Figure 4D and Table 2). The co-index may be used as a tool to identify patients with AA at both rs894151 and rs12438080 who, despite having HCC beyond Milan criteria, have an acceptable outcome profile (Figure 4E). Therefore, incorporation of tumor genetic variations into selection algorithms for LT candidates is a promising way to extend Milan criteria and allow more HCC patients to benefit from LT.

SNP rs894151 is intergenic between the pleckstrin homology domain-containing family F member 2 (PLEKHF2) and chromosome 8 open reading frame 37 (C8orf37) in chromosome 8q22. PLEKHF2 encodes an endoplasmic reticulum (ER)-associated protein. Overexpression of PLEKHF2 enhances tumor necrosis factor (TNF)-α-induced cellular apoptosis through an ER-mitochondrial apoptotic pathway [53]. In 15q26, rs12438080 lies on the longevity assurance homolog 3 (LASS3) gene, which is evolutionarily conserved from yeast to mammals [54] and encodes a ceramide synthase. 8q22 was reported to be associated with elevated expression of the metastasis gene metadherin (MTDH) with poor clinical outcomes in breast cancer [55]. Amplification of 15q26 in gastric cancer cell lines was associated with an up-regulated negative regulator of cell-cell adhesion [56]. Genome copy-number alteration and loss of heterozygosity in 15q26 were found in pediatric malignant astrocytomas [57] and breast cancer [58]. We genotyped healthy individuals and HBV infected patients to evaluate the distribution of genotypes on the two loci. We found the co-index of the two loci in either healthy group or HBV group showed significant difference from that in HCC group (Supplemental Text S1). Whereas, there was no difference between healthy group and HBV group. This result suggested that the two variations may result from acquired somatic mutations accumulating in the tumor genome.

RETRACTED

Patients with AG/GG at rs894151 have larger tumor sizes, increased tumor number and higher probability of microvessel invasion, while worse tumor differentiation was associated with AC/CC at rs12438080. The genetic variations of the two loci seem to represent the different features of the progression of HCC. Minor allele in the two loci may result in more aggressive tumor biologic behavior via interactions with neighboring tumor associated genes. Through this biologic change, HCC patients may get poorer prognosis after LT. However, the precise mechanism by which rs894151 and rs12438080 are associated with HCC recurrence and metastasis remains to be clarified and further investigated.

Like most studies focusing on organ transplantation, the sample size of this study is not very large, which made us to adopt a less stringent statistical cut-off for microarray analysis. And the sub-group analyses also came across this problem. This limitation predispose to a risk of false positive associations. Therefore, our result need to be further validated using a sufficiently large independent cohort from different transplantation centers. On the other hand, since the primary etiology of HCC in China is HBV infection, we do not have enough patients to be included in the study at that time. So, our study focused on HBV-related HCC. The prognostic value of the variation of the two loci shall be further evaluated for its clinical value across heterogeneous HCC patients, such as HCV-related or alcohol-related HCC, and Nonalcoholic steatohepatitis-related HCC.

In conclusion, the present study suggests that HBV-related HCC patients with allele G at rs894151 and/or C at rs12438080 in pretransplant plasma circulating DNA may bear an increased risk for HCC recurrence after LT. In contrast, patients with AA at both rs894151 and rs12438080 may experience a low recurrence risk, even in HCC patients exceeding Milan criteria. Genetic variations of rs894151 and rs12438080 in pretransplant plasma circulating DNA from HCC patients may predict recurrence after LT.

RETRACTED

## Supporting Information

Figure S1 Pre-array quality control and distribution of genome-wide *p*-values. Pre-array quality control using Mapping PCR test, PCR products were visualized on 2% agarose gels. *Sty* and *Nsp* represent different restriction enzyme digestions. Samples with fragments >750 bp indicate good quality for microarray hybridization. **A**, samples passing PCR-based QC tests. **B**, sample 11203 failed the QC test. **C**, genome-wide *p*-values of the Cochran-Armitage trend test. After filtration, 230,802 SNPs were included for analysis. The chromosomal distribution of *P*-values from the trend test is shown. The blue horizontal line represents a threshold of 10^−3^ for suggestive significance: 30 SNPs were above the horizontal line. The inset shows the quantile-quantile (Q-Q) plots of the observed *p*-values for association.
(TIF)

Figure S2 Hierarchical clustering of selected SNPs. Each SNP value was assigned based on the number of minor alleles. **A**, Hierarchical clustering of 1272 SNPs with *P*<.01. Each row represents an individual SNP and each column represents an individual tumor sample. **B**, Hierarchical clustering of 30 SNPs with *P*<.001. Each row represents an individual tumor sample and each column represents an individual SNP. Patients can be separated into two groups (high-risk or low-risk groups) using 30 top SNPs. The high-risk group had a shorter overall survival time (**C**) and time to recurrence (**D**) than the low-risk group (*P*<.001).
(TIF)

Figure S3 Kaplan-Meier analysis for recurrence (**A**) and survival (**B**) of patients harboring different numbers of risk alleles. Patients possessing more risk alleles had a higher recurrent risk and shorter survival time. The prognostic significance was assessed using Kaplan-Meier survival estimates and log-rank tests.
(TIF)

Table S1 Clinicopathological characteristics of three cohorts of HCC patients.
(DOC)

Table S2 Differences in allele frequencies between recurrence and non-recurrence groups in Training Set 2 (N = 102).
(DOC)

Table S3 Correlation between rs894151, rs1248080, and clinicopathological characteristics in Training Set (N = 102).
(DOC)

Table S4 Pairwise comparisons of TTR between patients with 0, 1, 2, and 3 risk alleles.
(DOC)

Table S5 Pairwise comparisons of OS between patients with 0, 1, 2, and 3 risk alleles.
(DOC)

Table S6 Univariate and multivariate analyses of factors associated with TTR in Validation Set (N = 77).
(DOC)

Table S7 AUC of the co-index and other factors.
(DOC)

Table S8 Clinicopathological characteristics of HCC patients beyond Milan criteria.
(DOC)

Table S9 Kaplan-Meier survival estimates and log-rank tests of factors associated with TTR and OS in patients exceeding UCSF criteria.
(DOC)

Table S10 Kaplan-Meier survival estimates and log-rank tests of factors associated with TTR and OS in patients within UCSF criteria.
(DOC)

Table S11 Univariate and Multivariate analyses of factors associated with tumor-related death in Training Set.
(DOC)

Text S1 Supporting information for methods and analysis.
(DOC)
